This article has been retracted.

# Propofol Prevents Autophagic Cell Death following Oxygen and Glucose Deprivation in PC12 Cells and Cerebral Ischemia-Reperfusion Injury in Rats

**DOI:** 10.1371/journal.pone.0035324

**Published:** 2012-04-11

**Authors:** Derong Cui, Li Wang, Aihua Qi, Quanhong Zhou, Xiaoli Zhang, Wei Jiang

**Affiliations:** 1 Department of Anesthesiology, Shanghai Sixth People's Hospital Affiliated with Shanghai Jiaotong University, Shanghai, China; 2 Department of Postgraduate School, Soochow University, Suzhou, China; Massachusetts General Hospital, United States of America

## Abstract

**Background:**

Propofol exerts protective effects on neuronal cells, in part through the inhibition of programmed cell death. Autophagic cell death is a type of programmed cell death that plays elusive roles in controlling neuronal damage and metabolic homeostasis. We therefore studied whether propofol could attenuate the formation of autophagosomes, and if so, whether the inhibition of autophagic cell death mediates the neuroprotective effects observed with propofol.

**Methodology/Principal Findings:**

The cell model was established by depriving the cells of oxygen and glucose (OGD) for 6 hours, and the rat model of ischemia was introduced by a transient two-vessel occlusion for 10 minutes. Transmission electron microscopy (TEM) revealed that the formation of autophagosomes and autolysosomes in both neuronal PC12 cells and pyramidal rat hippocampal neurons after respective OGD and ischemia/reperfusion (I/R) insults. A western blot analysis revealed that the autophagy-related proteins, such as microtubule-associated protein 1 light chain 3 (LC3-II), Beclin-1 and class III PI3K, were also increased accordingly, but cytoprotective Bcl-2 protein was decreased. The negative effects of OGD and I/R, including the formation of autophagosomes and autolysosomes, the increase in LC3-II, Beclin-1 and class III PI3K expression and the decline in Bcl-2 production were all inhibited by propofol and specific inhibitors of autophagy, such as 3-methyladenine (3-MA), LY294002 and Bafilomycin A1 (Baf),. Furthermore, in vitro OGD cultures and in vivo I/R rats showed an increase in cell survival following the administration of propofol, as assessed by an MTT assay or histochemical analyses.

**Conclusions/Significance:**

Our data suggest that propofol can markedly attenuate autophagic processes via the decreased expression of autophagy-related proteins in vitro and in vivo. This inhibition improves cell survival, which provides a novel explanation for the pleiotropic effects of propofol that benefit the nervous system.

## Introduction

Propofol is a widely used intravenous anesthetic. In addition to its sedation/hypnotic properties, propofol displays neuroprotective effects [1]–[3]. As an activator of GABA_A_ receptors, an inhibitor of NMDA receptors and a modulator of calcium influx through slow calcium channels, propofol improves the neurological outcome. In a rat cerebral ischemia model, propofol treatment was shown to decrease the infarct size in the hippocampus [4]. In addition, propofol administration also decreased the apoptotic rate and improved cell viability in hypoxic neuronal cultures [2], [3]. Moreover, propofol has a phenolic hydroxyl (OH) group, which is similar to that of vitamin E (α-tocopherol) and demonstrates antioxidant activity by scavenging free radicals [5], [6]. On the organelle and tissue level, the treatment of rat brain oxidative stress injury with propofol confers neuroprotective effects through an inhibition of lipid peroxidation [7]. Although, such pleiotropic mechanisms have been suggested to contribute to propofol-mediated neuroprotection, its capabilities are still not completely understood.

Recent evidence suggests that autophagy is activated in the pyramidal neurons of the rat hippocampus upon ischemic insult [8]–[10]. Autophagy is an evolutionarily conserved and highly regulated homeostatic process by which cytoplasmic macromolecules and organelles are degraded for removal or turnover through the lysosomal system [8]. However, excessive autophagy results in neuronal cell damage [8], [9]. The involvement of autophagy in neurodegenerative disorders is demonstrated by increased autophagic vacuoles [8], [9], with associated high levels of Beclin-1-phosphatidylinositol-3 kinase class III (class III PI3K) lipid-kinase-Vps34 and low levels of anti-apoptotic cellular Bcl-2 in pathological settings [11].

Apoptosis has been implicated in the delayed neuronal death induced by ischemia and has been extensively studied [12], [13]. However, autophagy could also mediate the execution of ischemia/reperfusion (I/R) injury-induced neuronal cell death, particularly in the hippocampus [8]–[10]. Therapies developed to target autophagy might have a beneficial effect on brain I/R injury.

Given the pleiotropic effects of propofol on nervous system function, we investigated the role of autophagy in propofol-mediated neuroprotection in vitro and in vivo. Our results are the first to show propofol-attenuated autophagic cell death in hypoxic neuronal PC12 cells and the rat hippocampus after I/R insult.

## Results

### Activation of Autophagy in Neuronal PC12 Cells after OGD Injury

In vitro ischemia was induced in cultured neuronal PC12 cells by OGD, which is a condition used to mimic in vivo metabolic inhibition [14]. Transmission electron microscopy was used to identify ultrastructural changes in neuronal PC12 cells at 0.5, 1, 3, 6 and 12 h after OGD insult. The control cells contained organelles, nuclei and chromatin with normal morphologies (Fig. 1AA). At 0.5–6 h after OGD, the PC12 cells contained many vesicles with the typical morphological features of autophagosomes. A number of isolated double or multi-membrane structures, which engulfed cytoplasmic fractions and organelles, were observed in the cytoplasm (Fig.1AB–AF, as indicated by the broad arrows).

**Figure 1:** Ultrastructural changes in PC12 cells after OGD injury. (A) The PC12 cells were subjected to OGD for 0.5 (AB), 1 (AC), 3 (AD), 6 (AE) and 12 h (AF) and were fixed for TEM examination. TEM micrograph features: Typical cytoplasms and nuclei in the control cells (AA, normal mitochondria indicated by black arrowheads). Isolated membrane and double- or multi-membrane autophagosomes in the PC12 cells following OGD treatment (AB–AF, as indicated by broad arrows). The mitochondria displayed swelling, dilation and cristae disruption (AB, AD and AE, as indicated by black arrowheads). The lysosomes were darkly stained, indicating the activation of lysosomes (AF, as indicated by narrow arrows). Cell shrinkage, nuclear condensation, loss of cellular organelles and vacuolization (AE and AF). N, nucleus; Broad arrows represent autophagosomes; Narrow arrows represent lysosomes; Black arrowheads represent mitochondria; Scale bar  =  1 µm. (B) Quantitative analysis of the number of intact mitochondria, autophagosomes and lysosomes in the OGD and control groups. Three samples in each group and ten fields for each sample were examined. The results are expressed as the mean ± SD. Statistical comparisons were conducted using an ANOVA followed by the Tukey test. *p <0.05 vs. control group.

A quantitative analysis of the cytoplasmic components showed a significant increase in the number of autophagosomes at 1–3 h after OGD (Fig. 1B). When the autophagosomes fused with the lysosomes, their inner membranes disappeared, and the autophagosomes became single-membrane autophagic vacuoles at 6–12 h after OGD (Fig.1AE and AF, as indicated by the broad arrows). The mitochondria displayed swelling, dilation and cristae disruption (Fig. 1AD and AE, as indicated by the black arrowheads), and the number of intact mitochondria was drastically decreased in a time-dependent manner (Fig. 1B). The lysosomal staining was darkened (Fig. 1AF, as indicated by the narrow arrows), and the number of lysosomes was obviously increased at 6 h after OGD (Fig. 1B), indicating the activation of lysosomes. Moreover, morphological features of apoptosis (Fig. 1AE) and necrosis (Fig. 1AF), such as cell shrinkage, chromatin condensation and damaged organelles with deteriorated membranes, were also observed at 12 h after OGD.

### Increased Expression of Autophagy-related Proteins in PC12 Cells Following OGD

Class III PI3K has been previously shown to activate autophagy, although the precise contribution of this specific substrate kinase to the regulation of LC3-II elevation under different cellular contexts is unclear. Our findings revealed that the class III PI3K pathway is involved in LC3-II upregulation, which promotes autophagy. The results demonstrated that the protein levels of class III PI3K were significantly upregulated and peaked at 1 h after OGD (Fig. 2A and C).

**Figure 2:** Increased class III PI3K (A and C), Beclin-1 (B and D), Bcl-2 (E and G) and LC3-II (F and H) expression in PC12 cells after OGD injury. PC12 cells were cultured, and OGD was induced as described in the methods. The cells were harvested for western blot analysis at various times after OGD. The optical densities of the respective protein bands were analyzed using Sigma Scan Pro 5 and normalized to the loading control (GAPDH). The results are expressed as the mean ± SD from three independent experiments. Statistical comparisons were conducted using an ANOVA followed by the Tukey test. *p < 0.05, **p < 0.01 vs. control group.

Beclin-1, a homologue of yeast Atg6, forms a protein complex with PI3K within the autophagosome [15]. The results demonstrated that the protein levels of Beclin-1 were significantly upregulated and peaked at 3 h after OGD (Fig. 2B and D).

Bcl-2 is an important anti-apoptotic protein. Previous studies have shown that excitotoxic and ischemic insults result in an autophagy-dependent decrease of Bcl-2 protein levels [8], [16]. As shown in Figure 2E and G, a marked reduction in Bcl-2 protein levels was observed 3 h following OGD treatment.

LC3 is required for the formation of autophagosome membranes [17]. The cytoplasmic form of LC3 (LC3-I) is diffusely distributed in the cytoplasm [18]. but is modified and concentrated in the autophagosomes during autophagy activation [17], [19]. When associated with autophagosomes, LC3 typically exhibits a shift in electrophoretic mobility from 18 to 16 kDa and is commonly referred to as LC3-II [17]. LC3-II is a common marker of autophagosomes in mammalian cells [17]. As shown in Figure 2, a dramatic increase in the LC3-II/LC3-I ratio was observed in PC12 cells 3 h after OGD treatment (Fig. 2F and H).

### Propofol Reduced the OGD-induced Cell Death

To determine the influence of propofol on OGD-induced cell injury, PC12 cells were treated with propofol or 3-MA during OGD. A concentration of 20–50 µmol/L of propofol or 20 mmol/L of 3-MA [8] effectively blocked the activation of autophagy, as evidenced by the inhibition of LC3-II production (Fig. 3A and B).

**Figure 3:** PC12 cells were treated with propofol (10, 20, 50 µmol/L) and 3-MA 20 mmol/L) during OGD treatment, and the cells were harvested 6 h later. (A) Immunoblotting LC3 in PC12 cells after OGD. Propofol at concentrations of 20 and 50 µmol/L and 3-MA at a concentration of 20 mmol/L effectively blocked the activation of autophagy, as evidenced by inhibiting the production of LC3-II. (B) The optical densities of the respective protein bands were analyzed using Sigma Scan Pro 5 and normalized to the loading control (GAPDH). The results are expressed as the mean ± SD from six independent experiments. Statistical comparisons were conducted using an ANOVA followed by the Tukey test. **p < 0.01 vs. control group; ^#^ *p* < 0.05 vs. OGD-treated group.

Lactate dehydrogenase (LDH) leakage was measured as an indicator of OGD-induced injury in PC12 cells [20]. The results showed that LDH leakage was markedly increased at 6 h after OGD. Propofol treatment resulted in a small but significant decrease in LDH leakage in a dose-dependent manner (Fig. 4A). Bafilomycin A1 (Baf) is a selective inhibitor of vacuolar H^+^-ATPase and therefore inhibits the maturation of autophagosomes. The results of the present study showed that the PC12 cell viability was decreased sharply 6 h after OGD. Propofol treatment significantly increased the cell viability of PC12 cells in a dose-dependent manner (Fig. 4B).

**Figure 4:** Inhibition of autophagy reduced OGD-induced PC12 cell injury. (A) Inhibition of OGD-induced lactate dehydrogenase (LDH) leakage by propofol and 3-MA. PC12 cells were treated with propofol (10, 20, 50 µmol/L) or 3-MA (20 mmol/L) during OGD treatment, and the cells were harvested 6 h later. Supernatants and cell lysates were prepared as described in the methods. LDH leakage was detected with a LDH assay kit according to the manufacturer’s protocol. The results are presented as the mean ± SD from three independent experiments. Statistical comparisons were conducted using an ANOVA followed by the Tukey test. (B) Inhibition of the OGD-induced reduction in PC12 cell viability by Baf. The PC12 cells were treated with various doses of propofol (10, 20 or 50 µmol/L) and Baf (4 µmol/L) for the indicated time, and cell viability was analyzed with an MTT assay. The results are presented as the mean ± SD from three independent experiments. Statistical comparisons were conducted using an ANOVA followed by the Tukey test. **p < 0.01 vs. control group; ^##^ *p* < 0.01 vs. OGD-treated group.

### The Effect of Propofol on the Expression of Autophagy-related Proteins in PC12 Cells Following OGD

Autophagy is primarily regulated by one central pathway: the class III PI3K-Beclin-1-Bcl-2-dependent mechanism. To explore how propofol regulates OGD-induced autophagy, we analyzed the expression of several autophagy-related proteins involved in this pathway in the OGD-injured PC12 cells. OGD injury resulted in a significant increase of Beclin-1 and LC3-II expression as compared with the control group (Fig. 5B, D, F and H). In addition, class III PI3K, which positively mediates autophagy, was greatly upregulated in the OGD-injured PC12 cells. However, treatment with propofol and/or LY294002 significantly decreased Beclin-1 and class III PI3K expression in PC12 cells (Fig. 5A–D), suggesting that OGD-induced autophagic cell death is dependent on the formation of the class III PI3K sub-complex containing Beclin-1.

**Figure 5:** Blockade of the inhibition of autophagy activation by propofol. PC12 cells were treated with propofol and the class III PI3K relatively selective inhibitor LY294002 (50 µmol/L) during the OGD insult and were harvested 6 h later for western blot analysis. (A, B, E, F) Immunoblot analyses of OGD-injured PC12 cells. The PC12 cell homogenates were analyzed by western blotting using a specific antibody against each autophagy-related protein. The expression of GAPDH was also examined for the protein loading control. (C, D, G, H) Quantification of class III PI3K, Beclin-1, Bcl-2, LC3-I and LC3-II expression. Each protein (class III PI3K,class III PI3K, Beclin-1, Bcl-2, LC3-Ι and LC3-II) shown in Fig. 5A, B, E, F was quantified after a densitometric scan and normalized to GAPDH. The optical densities of the respective protein bands were analyzed using Sigma Scan Pro 5 and normalized to the loading control (GAPDH). The results are expressed as the mean ± SD from three independent experiments. Statistical comparisons were conducted using an ANOVA followed by the Tukey test. **p < 0.01 vs. control group; ^#^ *p* < 0.05, ^##^ *p* < 0.01 vs. OGD-treated group.

To further confirm the influence of propofol on the response of the class III PI3K-Beclin-1-Bcl-2 interaction to OGD-induced autophagy in the presence of propofol, the cells were transiently transfected with small interference RNA (siRNA) against Beclin1 for 0–72 h (Fig. 6A, B), which is a principal regulator in the formation of autophagosomes and the initiation of autophagy through the class III PI3K pathway or the inhibition of autophagy through the Bcl-2 pathway. We observed a significantly increased interaction between Beclin-1 and class III PI3K, leading to Beclin-1-dependent autophagic cell death, while the administration of propofol promoted Bcl-2 protein expression and significantly decreased class III PI3K protein expression in the OGD-injured PC12 cells (Fig. 5A, C, E, G and Fig. 7A-F). These observations suggest that the decreased expression of Beclin-1 and class III PI3K or the increased Bcl-2 expression by propofol in the OGD-injured PC12 eventually inhibits autophagy.

**Figure 6:** PC12 cells were transfected with Beclin-1 siRNA at specific concentration (100 nM) for various times. (A) The inhibition of Beclin-1 protein expression by siRNA transfection was measured by immunoblot assay with an anti-Beclin-1 antibody. GAPDH was used as the loading control. (B) Quantification of Beclin-1 expression. The Beclin-1 protein shown in Fig. 6A was quantified after a densitometric scan and normalized to GAPDH. The optical densities of the respective protein bands were analyzed using Sigma Scan Pro 5 and normalized to the loading control (GAPDH). The results are expressed as the mean ± SD from three independent experiments. Statistical comparisons were conducted using an ANOVA followed by the Tukey test. *p < 0.05, **p < 0.01 vs. 0 hour group.

**Figure 7:** The expression of autophagy-related proteins during 6 h of OGD after transfection with Beclin-1 siRNA at specific concentration (100 nM) for 48 h. (A, B, E) Immunoblot analyses of OGD-injured PC12 cells. The PC12 cell homogenates were analyzed by western blotting using a specific antibody against each autophagy-related protein. The expression of GAPDH was also examined as the protein loading control. (C, D, F) The quantification of class III PI3K, Bcl-2, LC3-I and LC3-II expression. Each protein (class III PI3K, Bcl-2, LC3-I and LC3-II) shown in Fig. 7A, B, E was quantified after a densitometric scan and normalized to GAPDH. The optical densities of the respective protein bands were analyzed using Sigma Scan Pro 5 and normalized to the loading control (GAPDH). The results are expressed as the mean ± SD from three independent experiments. Statistical comparisons were conducted using an ANOVA followed by the Tukey test. *p < 0.05, **p < 0.01 vs. the 0 hour group.

### The Injury of Hippocampal Pyramidal Neurons Following I/R

Studies have reported an early decline in the number of hippocampus CA1 pyramidal neurons following severe ischemic insults [13], [21]. To specifically investigate the temporal effects of I/R on hippocampal pyramidal neuron function, we measured the number of pyramidal neurons in the CA1 region of the hippocampus following severe ischemic insults at various time points using histochemical techniques. The results revealed that, as compared with the control group (Fig. 8A), there was no robust change in the number of hippocampal pyramidal neurons at 1 h after ischemia (Fig. 8B). This result was consistent with the observation the lack of LC3 expression in the CA1 hippocampus at that time point (Fig. 9A). However, the number of hippocampal pyramidal neurons was reduced in the ischemic CA1 hippocampus at 3 h (Fig. 8C) and was further decreased at 6–24 h after ischemia (Fig. 8D, E and F). Moreover, the damaged pyramidal neurons in the ischemic CA1 hippocampus exhibited various stages of fragmentation (Fig. 8F), which is characteristic of dying cells, indicating that the hippocampal pyramidal neurons were damaged and died in a time-dependent manner following I/R.

**Figure 8:** The neuronal damage and histological characteristics of necrotic neurons were assessed by a histological examination. Thionine staining of brain sections at the level of the hippocampus from sham (*n* = 6) rats and rats sacrificed at 1, 3, 6, 12, or 24 h after I/R (*n* = 6 per time point). (A) Sham brain sections revealed normal neurons in the hippocampus. (B–C) Sections from 1 h and 3 h after a 10-min period of brain ischemia showed neuronal loss, and a small number of neurons in the CA1 area exhibited the morphological criteria of necrosis, displaying cell shrinkage, nuclear condensation, and fragmentation. (D–F) A dramatic loss of neurons was observed in the CA1 cell layer at 6, 12, and 24 h after ischemia. (H) Quantitative analysis of the number of pyramidal neuronal cells. The number of pyramidal neurons in the ischemic hippocampus was significantly decreased in the ischemic rats compared to the sham rats. The data are expressed as the percentage of sham-operated group animals and as the mean ±SD, *n* =  6. The statistical analysis was performed using a one-way ANOVA. *p < 0.05, **p < 0.01 vs. sham group. Scale bars: lower magnification (G), 50 µm; higher magnification (A-F), 500 µm. so, stratum oriens; sp, stratum pyramidal; sr, stratum radiatum.

We also measured the expression of LC3 ΙΙ by immunohistochemistry at various time points following the ischemic insult (Fig. 9A). LC3 ΙΙ is a marker for autophagic vacuoles (AVs). When the hippocampal pyramidal neurons were examined by fluorescence microscopy after I/R treatment, the immunohistochemistry-labeled AVs appeared as distinct puncta distributed throughout the cytoplasm, the perinuclear regions and the processes. As compared with the control group (Fig. 9A), there was a significant increase in the number of LC3 II-labeled vesicles at 1 h (Fig. 9A and B), which peaked at 3–6 h after I/R treatment (Fig. 9A and B), suggesting an induction of AV formation in hippocampal pyramidal neurons after I/R.

**Figure 9:** LC3-II was detected with a monoclonal anti-LC3-II-FITC antibody (green). The sections were taken from the infarct regions of the ipsilateral hippocampus 1, 3, 6, 12 and 24 h following I/R. I/R increased the LC3-II-positive cells and LC3-II protein levels in the ischemic hippocampus after I/R in rats. I/R was induced by two-vessel occlusion. Representative photomicrographs of LC3-II immunofluorescence. Immunofluorescence of LC3-II was performed at 0–24 h after I/R. Images (magnification 200x) were taken from the same part of the ischemic hippocampus. (B) The quantitative analysis of the number of LC3-II-positive cells. The number of LC3-II-positive cells in the ischemic hippocampus was significantly increased in the ischemic rats compared to the sham rats. The data are expressed as percentage of the sham-operated animals and as the mean±SD, *n*  =  6. The statistical analysis was performed using a one-way ANOVA. *p < 0.05, **p < 0.01 vs. sham group.

### Activation of Autophagy in Rat Hippocampal Pyramidal Neurons after I/R

The ultrastructural changes in rat hippocampal pyramidal neurons were observed by transmission electron microscopy at 1–24 h after I/R. The smooth cytoplasmic, normal appearance of the mitochondria (Fig. 10AA, as indicated by black arrowheads), nuclei and chromatin were observed in the control hippocampal pyramidal neurons. After the I/R insult, the pyramidal neurons exhibited typical signs of autophagic/lysosomal activation and apoptosis, as shown in Figure 10AB–AF. Autophagosomes were observed as C-shaped double membrane structures or double membrane vacuoles (Fig. 10AB–AF, as indicated by broad arrows). The most abundant autophagosomes were observed at 3 h after I/R (Fig. 10C and G). Occasionally, autophagosomes with engulfed organelles were observed. The fusion of autophagosomes with lysosomes was occasionally observed (Fig. 10AD, as indicated by asterisks). The mitochondria displayed swelling, dilation and cristae disruption (Fig. 10AC, AD and AE, as indicated by black arrowheads), and the number of intact mitochondria were dramatically decreased in a time-dependent manner (Fig. 9G). Lipid drops were phagocytized by lysosomes that were darkly stained (Fig. 10AD and as indicated by narrow arrows), and the quantitative analysis of the change in numbers of lysosomes also showed that the number of lysosomes was markedly increased 6 h after I/R (Fig. 10G), indicating the activation of lysosomes. The loss of organelles and cytoplasm vacuolization was apparent 6 h after the I/R insult (Fig. 10AD). In addition, both apoptotic and necrotic morphological features were observed in the same cell; e.g., cell shrinkage, large chromatin clumping, nuclear condensation/fragmentation, swollen cytoplasm, damaged organelles and deteriorated membranes were observed in the same pyramidal neurons at 24 h after I/R (Fig. 10AF). The quantitative analysis of the cytoplasmic components also revealed that the number of lysosomes was markedly increased at 6 h after I/R (Fig.10B), indicating the activation of lysosomes.

**Figure 10:** Ultrastructural changes in rat hippocampal pyramidal neurons at 1 (AB), 3 (AC), 6 (AD), 12 (AE) and 24 h (AF) after I/R. (A) Transmission electron microscopy (TEM) images showing: the normal appearance of the cytoplasms, organelles and nuclei in the control hippocampal pyramidal neurons (AA, normal mitochondria indicated by black arrowheads); C-shaped double-membrane structures and double-membrane autophagosomes in the hippocampal pyramidal neurons following I/R treatment (AB–AF, as indicated by broad arrows); swelling, dilation and cristae disruption in mitochondria (AC, AD and AE, as indicated by black arrowheads); and activated lysosomes (AD, as indicated by narrow arrows). An autophagosome fused with a lysosome (AD, as indicated by an asterisk). The coexistence of morphological features of necrosis and apoptosis in the same neurons (AF). N, nucleus; Broad arrows represent autophagosomes; Narrow arrows represent lysosomes; Black arrowheads represent mitochondria; Asterisks represent autolysosomes. Scale bar  =  1 µm. (B) The quantitative analysis of the number of intact mitochondria, autophagosomes and lysosomes in the ischemic and control groups. Three rats in each group and 10 fields for each rat were examined. The results are expressed as the mean ± SD. The statistical comparisons were conducted using an ANOVA followed by the Tukey test. *p < 0.05 vs. control group.

### Propofol Reduced the I/R-induced Death of Cells

To further address the function of propofol in the cerebral ischemia-induced damage of hippocampal pyramidal neurons in vivo, we examined the effects of propofol (i.p., 10, 50, and 100 mg/kg ) or 3-MA (i.c.v., 600 nmol) on the number of CA1 hippocampus pyramidal neurons using histochemical techniques and the number of LC3 II-positive cells using immunofluorescence at 12 h after I/R. The results showed that the number of pyramidal neurons in the ischemic pyramidal layers of the CA1 hippocampus was dramatically decreased, and the number of LC3 II-positive cells was dramatically increased, in the ischemic rats (Fig. 11B). In contrast, propofol (i.p., 50 and 100 mg/kg) or 3-MA significantly increased the number of pyramidal neurons and decreased the number of LC3 II-positive neurons (Fig. 11A). These results suggest persistent and excessive autophagy/lysosome activation induced by the in vivo ischemia of pyramidal neurons, and the inhibition of autophagy by propofol mildly increased cell survival.

**Figure 11:** Propofol increased the number of the hippocampal pyramidal neurons and decreased the expression of the LC3-II protein and the number of lysosomes and autophagosomes in the ischemic hippocampus after I/R in the rats. I/R was induced by 2-vessel occlusion. Propofol 10, 50, or 100 mg/kg was administrated intraperitoneally and 3-MA (600 nM) was administered intracerebroventricularly 10 min after the onset of ischemia. (1) Sham-operated group (control group, Cont); (2) I/R group; (3) I/R+ 3-MA 600 nmol group; (4) I/R + propofol 10 mg/kg group; (5) I/R + propofol 50 mg/kg group; (6) I/R + propofol 100 mg/kg group; (7) I/R + vehicle (intralipid, 100 mg/kg) group. Histochemical, immunohistochemical and TEM morphological analyses were performed at 12 h after I/R. (A) Quantitative analysis of the number of hippocampal pyramidal neurons. The number of hippocampal pyramidal neurons in the ischemic hippocampus was significantly increased in the propofol- and 3-MA treated rats, compared to the ischemic rats. (B) Quantitative analysis of the number of LC3-II-positive neurons. The number of LC3-II-positive neurons in the ischemic hippocampus was significantly decreased in the propofol- and 3-MA treated rats compared to the ischemic rats. The data are expressed as percentage of the sham-operated animals and as the mean±SD, *n*  =  6. Statistical analyses were performed using a one-way ANOVA. **p < 0.01 vs. control group; ^##^ *p* < 0.01 vs. I/R-treated group. (C) Quantitative analysis of the number of intact mitochondria, autophagosomes and lysosomes in the ischemic group, the propofol- or 3-MA treated group and the control group. Six rats in each group and 10 fields for each rat were examined. The results were expressed as the mean ± SD. Statistical comparisons were conducted using an ANOVA followed by the Tukey test. *p < 0.05 vs. control group. #*p* < 0.05 vs. I/R-treated group.

Quantitative analysis of the number of intact mitochondria, autophagosomes and lysosomes in the ischemic model, propofol-treated, 3-MA-treated and control groups (Fig 11C) revealed that the number of autophagosomes and lysosomes in the ischemic hippocampus was dramatically increased, and the number of was intact mitochondria was dramatically decreased in the ischemic rats. In contrast, the administration of propofol (i.p., 50 and 100 mg/kg) or 3-MA significantly decreased the number of autophagosomes and lysosomes and increased the number of intact mitochondria.

There were no significant changes in the pH, the arterial carbon dioxide (PaCO_2_) or oxygen (PaO_2_) concentrations or blood glucose concentrations before and after the intracerebral ventricular injection of 3-MA or the intraperitoneal injection of propofol in any of the groups (Table 1).

**Table 1:** Physiological parameters.

Groups	Time	MAP(mmHg)	PH	PaCo_2_(mmHg)	Po_2_(mmHg)	GI(mg/dl)
Cont	Baseline	105±6	7.38±0.02	35.6±2.9	146.2±18.2	156±23
	Ischemia	103±5	7.43±0.03	36.8±2.8	141.5±19.3	166±16
	Recovery	107±5	7.37±0.03	38.5±2.2	140.5±13.2	165±21
I/R	Baseline	105±6	7.40±0.02	38.3±2.6	144.3±11.8	158±22
	Ischemia	39±3^a^	7.42±0.03	36.9±2.8	136.6±16.5	161±19
	Recovery	110±5	7.39±0.03	39.3±3.2	139.8±19.2	163±18
I/R+3-MA(600nM)	Baseline	105±6	7.37±0.02	38.3±3.1	138.6±15.5	165±18
	Ischemia	41±2^a^	7.43±0.03	38.6±2.3	143.3±16.8	155±19
	Recovery	116±4	7.39±0.02	38.9±3.1	140.3±18.3	158±21
I/R+Prop(10mg/kg)	Baseline	105±6	7.39±0.03	37.8±2.6	142.3±16.9	163±20
	Ischemia	38±3^a^	7.41±0.02	38.5±2.5	143.5±18.6	159±18
	Recovery	113±6	7.43±0.03	39.5±2.1	141.6±16.2	156±17
I/R+Prop(50mg/kg)	Baseline	108±3	7.39±0.03	38.6±3.3	143.3±18.3	159±16
	Ischemia	39±2^a^	7.41±0.01	39.6±3.8	143.5±16.5	160±15
	Recovery	115±6	7.42±0.03	40.5±2.3	143.3±11.5	161±18
I/R+Prop(100mg/kg)	Baseline	105±6	7.39±0.02	39.6±2.9	141.6±18.5	162±16
	Ischemia	41±3^a^	7.39±0.02	40.8±3.1	142.6±16.9	169±15
	Recovery	110±4	7.42±0.03	39.8±2.6	144.3±12.8	168±19
I/R+Int(100mg/kg)	Baseline	105±6	7.38±0.02	40.3±3.2	143.6±15.8	173±18
	Ischemia	39±2^a^	7.41±0.03	39.9±2.8	143.8±18.5	169±26
	Recovery	113±5	7.42±0.01	38.9±2.1	140.9±16.9	165±21

All values are mean±SD. Arterial blood gas tensions include PaO_2_, PaCO_2_, PH and GI.

MAP, mean arterial pressure; PaO_2_, arterial oxygen pressure; PaCO_2_, arterial carbon dioxide pressure; GI, glucose.

a Controlled parameter.

### Effect of Propofol on the Expression of Autophagy-related Proteins During I/R

The brain I/R injury resulted in a significant increase in Beclin-1 and LC3-II expression as compared with the control group (Fig. 12B, D, F, H). In addition, class III PI3K, which positively mediates autophagy, was greatly upregulated in the I/R-injured brains. However, the administration of propofol significantly increased Bcl-2 expression and prevented I/R-dependent Beclin-1and class III PI3K protein expression after I/R injury (Fig. 12A-D, E, G). The western blot analysis showed a decreased conversion of LC3-I to LC3-II in the hippocampi of the propofol-treated group at 12 hours after I/R injury (Fig. 12F, H).

**Figure 12:** Inhibition of autophagy activation by propofol. I/R was induced by 2-vessel occlusion. Propofol 100 mg/kg was administrated intraperitoneally and 3-MA (600 nM) was administered intracerebroventricularly 10 min after the onset of ischemia. The rats were treated with propofol (100 mg/kg) and the autophagy inhibitor 3-MA (600 nM) during the I/R insult and were sacrificed 12 h later for western blot analysis. (A, B, E, F) Immunoblot analyses of the I/R-injured hippocampus. The hippocampus homogenates were analyzed by western blotting using an antibody specific against each autophagy-related protein. The expression of GAPDH was also examined as the protein loading control. (C, D, G, H) The quantification of class III PI3K, Beclin-1, Bcl-2, LC3-I and LC3-II expression. Each protein (class III PI3K, Beclin-1, Bcl-2, LC3-I and LC3-II) shown in Fig. 12A, B, E, F was quantified after a densitometric scan and normalized to GAPDH. The optical densities of the respective protein bands were analyzed using Sigma Scan Pro 5 and normalized to the loading control (GAPDH). The results were expressed as the mean ± SD from six independent experiments. Statistical comparisons were conducted using an ANOVA followed by the Tukey test. **p < 0.01 vs. control group;^ ##^ *p* < 0.01 vs. I/R group.

## Discussion

The major findings of the present study are that propofol therapy achieves a greater inhibition of autophagic cell death in both in vitro and in vivo models of neuronal ischemia.

We demonstrated the positive effect of propofol on the inhibition of OGD-induced autophagosomes in neuronal PC12 cells. The formation of such autophagosomes is essential for autophagic cell death [8]–[10], as demonstrated by the increased numbers of LC3-II-positive neurons and the increased expression of class III PI3K and Beclin-1, which are key proteins in autophagy induction [22], [23].

The prevention of neuron death by the inhibition of autophagy after hypoxic-ischemic injury has been documented to be dependent on an autophagy induction-related gene, Atg7. The present results indicate that a group of factors including class III PI3K, Beclin-1 and Bcl-2 are also engaged in the neuroprotection of propofol against OGD-induced damage in neuronal PC12 cells. The experimental evidence supporting such an argument includes the inhibition of class III PI3K-Beclin-1, the formation of autophagosomes, and the increase in the level of Bcl-2 by propofol in vitro. The role of autophagy in neurodegeneration and neuroprotection is elusive. Rapamycin, an autophagy-inducing drug, can provide protection in models of neurodegenerative diseases [24], which indicates that neurodegeneration is inhibited by autophagy [25]. However, excessive autophagic responses could become hazardous and harmful. Indeed, it has been demonstrated that mutations in lysosomal surface proteins and a variety of deficits in lysosomal enzymes are able to cause prominent neurodegeneration. The results of the present study revealed that the formation of AVs in both OGD-exposed PC12 cells and I/R-injured hippocampal neurons in rats was associated with a reduced number of cells, indicating that autophagy-related processes may promote cell death. This result agrees with those of Li et al [26], who showed that the inhibition of autophagy with lithium reduced brain injury after hypoxia-ischemia in neonatal rats. The present data also indicate that autophagic cell death was attenuated by propofol, adding a new neuroprotective mechanism for this agent that has not been reported previously.

A number of mechanisms have been associated with the neuroprotective effects of propofol, including [27] the reduction in the cerebral metabolic rate of oxygen, the antioxidant-based removal of lipophilic and hydrophilic radicals [1], [5], the activation of γ-aminobutyric acid type A receptors [28], the inhibition of glutamate receptors [29], and the reduction of the extracellular glutamate concentrations by inhibiting Na^+^ channel-dependent glutamate release [30] or the enhancement of glutamate uptake [2], [31]. In this study, our results demonstrated that propofol significantly reduced the degree of cell damage induced by OGD injury in neuronal PC12 cells. We found that OGD-induced cell death is associated with the activation of autophagy through the expression of class III PI3K, Beclin-1 and LC3-II, and the accumulation of autophagic vacuoles. This autophagic cell death was inhibited by the administration of propofol through the reversal of the activation mechanism during OGD.

To further validate our findings in vitro, we used a two-vessel occlusion model in rats to induce brain injury because forebrain ischemia is often expected in a clinical setting. This model could imitate cerebral ischemia resulting from acute bleeding, cardiac arrest and certain types of shock [13]. In this study, our results demonstrated that propofol significantly reduced the degree of hippocampus damage induced by I/R injury in rats. In our I/R model, the neuroprotection of propofol was less effective than that reported in models of transient focal ischemia [4], [13]. This difference could be attributed to the model itself; our model is more severe because we used a single injection of propofol rather than continuous infusion. Additionally, propofol reduced the expression of class III PI3K and Beclin-1 and increased the expression of Bcl-2. Previous studies [32] found that the brain protective effect of propofol during I/R was mediated by the inhibition of Bcl-2 dissociation from Beclin-1, resulting in a significant decrease in autophagic cell death. The interaction of Beclin-1 with Bcl-2 was diminished by I/R injury and was rescued by propofol to levels comparable with those observed in the control. These results also suggested that propofol might modulate autophagy via class III PI3K-Beclin-1-Bcl-2 dependent pathways.

There are a number of issues in this study that still must be clarified. (1) Because we used a recovery interval of 12 or 24 h for PC12 cells exposed to OGD and for rats after I/R, we cannot exclude a transient neuroprotective effect for propofol, as reported for other anesthetics [33]. However, in an incomplete cerebral ischemia and reperfusion model, propofol offered long-term neuroprotection [34]. In addition, the early evaluation of the neuroprotective effects of propofol seem to indicate the long-term improvement of brain function in rats exposed to mild brain ischemia [7]. (2) The concentrations of propofol that were used in OGD-injured PC12 cells have been reported in previous publications [35], [36], but are considered to be high compared with the commonly used clinical concentration. The total amount of propofol administered in I/R rats was in accordance with the amount used in the study by Arcadi et al [37]. A single intraperitoneal injection of 50 or 100 mg/kg propofol could significantly attenuate CA1 injury after global ischemia in rats. These doses are also considered to be high. (3) It is still unclear how propofol directly modulates the expression of autophagy-related genes and the activation of lysosomes when the brain is exposed to the I/R injury. Therefore, further in vivo and in vitro studies focusing on the regulation of autophagy-related genes and lysosomal activation will contribute to the development of specific drugs that can be used to treat and/or prevent autophagy-mediated neuronal death. Despite these limitations, our study shows that propofol is neuroprotective in PC12 cells exposed to OGD in vitro, potentially through the inhibition of autophagy activation and maturation. In a severe model of forebrain cerebral ischemia in vivo, propofol reduces the extent of the injury of hippocampal pyramidal neurons and prevents ultrastructural changes.

In summary, the present results indicated that the negative effects of OGD and I/R, including the formation of autophagosomes and autolysosomes, the increases in LC3-II, Beclin-1 and class III PI3K expression and the decrease in Bcl-2 production were all inhibited by propofol. Furthermore, in vitro OGD cultures and I/R rats exhibited an increase in cell survival following the administration of propofol. These results also suggest that autophagy might represent a novel mechanism by which I/R damage induces cell death, and the inhibition of autophagy activation and maturation by propofol might reduce I/R injury in brain. Our findings suggest a novel strategy for the development of a novel therapy for damage due to brain hypoxia.

## Materials and Methods

### Preparation and Incubation of Neuronal PC12 Cells

Neuronal PC12 cells were obtained from the Key Laboratory of Neurobiology, Institute of Medicine, Shanghai Institutes for Biological Sciences, Chinese Academy of Sciences and cultured in RPMI 1640 medium (Gbico/Life Technologies Ltd, Paisley, Scotland) supplemented with 10% fetal bovine serum (Gibco/Life Technologies Ltd, Paisley, Scotland) and 7.5% horse serum (Gibco/Life Technologies Ltd, Paisley, Scotland) in a humidified incubator (Hira Sawa Work, Japan) at 37°C and 5% CO_2_. For the survival experiments, the PC12 cells were seeded (2–10^3^ cells/well) on 96-well plates in culture medium supplemented with 10 nM mouse 7S nerve growth factor (NGF) (Sigma, Saint Louis). After 3 days, additional NGF was added (10 nM). After 6 days of culture with NGF, more than 95% of the cells appeared to be morphologically differentiated with neurites at least twice the length of the cell body diameter; the cells were exposed to combined oxygen and glucose deprivation (OGD) at 0, 0.5, 1, 3, 6 and 12 h on the seventh day.

### Oxygen and Glucose Deprivation (OGD) Treatment and Assessment of PC12 Cells Injury

Combined oxygen and glucose deprivation (OGD) was performed as described previously [14], [38]. Briefly, ischemia was introduced by a buffer exchange to Hanks solution, which is an ischemia-mimetic solution (in mmol/L: 140 NaCl, 3.5 KCl, 0.43 KH_2_PO_4_, 1.25 MgSO_4_, 1.7 CaCl_2_, 5 NaHCO_3_, 20 HEPES, pH 7.2–7.4) and subsequently, the culture dishes were placed in a hypoxic incubator chamber (Billups-Rothenberg) equilibrated with 95% N_2_/5% CO_2_ at 37°C for 0.5, 1, 3, 6 and 12 h. The buffered Hanks solution was previously gassed with 95% N_2_/5% CO_2_ for 30 min. The control cells were incubated in RPMI 1640 medium solution and run in parallel for each condition for the indicated time periods corresponding to those of the experimental groups. Solutions of 10% Intralipid at a concentration of 50 µM (used as a vehicle control, Sigma, St Louis, MO) and propofol (10, 20 or 50 µM) (AstraZeneca UK Limited) were preincubated for 10 min before and during OGD stimulation. 3-MA (20 mM) (Sigma, 08592(fluka) [8], a specific inhibitor of autophagosome formation, was added as a positive control. For the western blot analysis of the effects of propofol on autophagy-related proteins, the PC12 cells were cultured in 60 mm dishes, harvested and probed for autophagy-related proteins after 0, 0.5, 1, 3, 6 and 12 h of OGD.

### Transmission Electron Microscopic Analyses of Autophagosomes in PC12 Cells after OGD Injury

The PC12 cells were cultured in 60 mm dishes and treated with OGD for 0.5, 1, 3, 6 and 12 h. After treatment, the cells were fixed with 4.0% paraformaldehyde in phosphate-buffered saline (PBS) and then post-fixed with 2.0% glutaraldehyde in 0.1 mol/L PBS and preserved at 4°C for further processing. When the processing resumed, the cells were post-fixed in 1% osmium tetroxide in PBS, dehydrated in graded alcohols, embedded in Epon 812, sectioned with an ultramicrotome, and stained with uranyl acetate and lead citrate. The sections were examined using a transmission electron microscope (Technai 10; Philips).

### Cytotoxicity Assay

Lactate dehydrogenase (LDH) leakage not only occurs during necrosis but also during apoptosis [39]. Because 3-MA interferes with the MTT assay, LDH leakage was assessed as an index of cell death after the PC12 cells were treated with OGD [20], [40]. To examine the contribution of propofol to the OGD-induced death of PC12 cells, the cells were treated with propofol (10, 20 or 50 µmol/L) and 3-MA (20 mmol/L) during OGD. LDH leakage was measured 6 h after OGD. Briefly, after OGD treatment, the supernatant of the cell culture was harvested. The PC12 cells were rinsed with PBS and lysed with 1% Triton X-100 at 37°C for 30 min. The supernatants and cell lysates were prepared following the manufacturer’s instructions for the LDH assay using a cell viability assay kit (Nanjing Jiancheng Bioengineering Institute, A020). The absorbance value (*A*) at 440 nm was determined with an automatic multiwell spectrophotometer (Bio-Rad Laboratories, Hercules, CA, USA). LDH leakage was calculated using the following formula: LDH leakage (%)  =  (*A* positive/*A* positive blank)/(*A* negative/*A* negative blank) × 100% [41].

### Cell Viability Assay

PC12 cell viability was determined with a 3-(4, 5-dimethylthiazol-2-yl)-2,5-diphenyltetrazolium bromide (MTT, Sigma, M5655use) assay 6 h after OGD treatment in accordance with a previously described method [42]–[44]. To examine the contribution of propofol to OGD-induced PC12 cell death, PC12 cells were treated with propofol (10, 20 or 50 µmol/L) and the autophagy inhibitor Bafilomycin A1 (Baf, 4 µmol/L, Alexis Biochemicals, Alx-380–030) during OGD. Briefly, the MTT solution was added to the culture medium (final concentration  =  500 µg/mL) at the end of the OGD treatment. The reaction was terminated by the addition of 10% acidified SDS (100 µL) to the cell culture 4 h after the MTT addition. The absorbance value (*A*) was measured at 570 nm using a multiwell spectrophotometer (Bio-Rad Laboratories). The percentage of cell death was calculated using the following formula: cell death (%) =  (1-*A* of experiment well/*A* of control well) × 100%.

### Assay of the Effects of Propfol on Autophagy-related Proteins

To confirm whether propofol blocks the autophagic process, the effects of propofol on autophagy-related proteins were assessed. The OGD time (6 h) and the final concentration of propofol (50 µM) were determined by pilot studies and the average blood propofol concentration during human brain surgery in our clinical project [6], [45]. For the inhibitory experiments, the cells were pre-incubated with a selective PI3K inhibitor (LY2940002, final concentration 50 µM, Cell Signaling Technology, #9901) for 10 min, and then treated with OGD and/or propofol or Intralipid. These drugs were diluted in serum-free medium prior to their addition to the cultures. The cells were randomized into seven groups: Group 1, control (untreated); Group 2, cells were subjected to 6 hours of OGD; Group 3, cells treated with OGD and propofol (50 µM); Group 4, cells treated with OGD and Intralipid (50 µM); Group 5, cells treated with OGD and LY294002 (50 µM, prepared 10 min prior to the OGD treatment); Group 6, cells treated with OGD and LY294002 (50 µM) and propofol (50µM); and Group 7, cells treated with OGD and LY294002 (50 µM) and Intralipid (50 µM). For the western blot analysis of the effects of propofol on autophagy-related proteins, the PC12 cells were cultured in 60-mm dishes and harvested after 6 h of OGD.

### Transfection of Cells with Beclin1 siRNA

The cells were transiently transfected with small interference RNA (siRNA) against Beclin-1 (Refseq number: NM-001034117, NM-053739; siRNA ID: 195717; Ambio INC, Austin, TX, USA), a principal regulator in the formation of autophagosomes and the initiation of autophagy through the PI3K class III pathway, using Lipofectamine™ 2000 (Invitrogen, Carlsbad, CA, USA). The cells transfected with siRNA #3 were used as a negative control. The transfected cells were randomized into four groups followed by immunoblot assay: Group 1, control (untreated); Group 2, subjected to 6 h of OGD; Group 3, treated with OGD and propofol (50 µM); and Group 4, cells treated with OGD and Intralipid (50 µM). For the western blot analysis of the effects of propofol on autophagy-related proteins, the PC12 cells were cultured in 60-mm dishes and harvested after 6 h of OGD.

### Animal and Surgical Protocol

Male Sprague-Dawley rats weighing approximately 250–300 g were purchased from the Experimental Animals Center of Shanghai Jiaotong University (certificate No. 201000082, Grade II) and surgically prepared for I/R injury as described previously [13]. All the procedures were performed in accordance with the Guide for Care and Use of Laboratory Animals published by the National Institutes of Health (Guide for the Care and Use of Laboratory Animals, 1996). The Animal Research Committee of Shanghai Jiaotong University in China approved the protocol.

All the rats were fasted for 8–12 h, and water was provided ad libitum; other conditions were constantly controlled. Anesthesia was induced in a Plexiglas chamber with 4% halothane; the animals were then tracheally intubated and mechanically ventilated with 1.5% halothane in 30% O_2_/70% N_2_O. No muscle relaxants were given during the anesthesia. The left femoral artery was cannulated to monitor the blood pressure and to collect the blood, and the right external jugular vein was used for drug administration and for blood reinjection. Digital thermistor probes (Multi-thermistor Meter D321; Technol Seven, Yokohama, Japan) were placed in the rectum to monitor the core temperature, which was maintained at 37±0.5°C using an electrically heated blanket. The arterial blood samples were collected for blood gas analysis after the isolation of the bilateral common carotid arteries from the carotid sheaths using a ventral midline incision. If the blood gas parameters were PO_2_ 90–140 mmHg, PCO_2_ 35–45 mmHg, pH 7.35–7.45, GI 150–180 mg/dl, cerebral ischemia was induced by clamping the common carotid arteries with small vascular clips and inducing hypotension (MAP: 40±5 mm Hg) by withdrawing and injecting blood for 10 min. Forebrain ischemia was confirmed by an EEG indicating the complete suppression of electroencephalographic activity. Thereafter, the clips were removed, and the withdrawn blood was reinfused. At the end of the anesthesia process, the vascular catheters were removed, and the wounds were sutured. The endotracheal catheter was extubated until there was a recovery of spontaneous respiration and the righting reflex.

Sham-operated rats underwent the same procedures, except for the I/R. To observe the time course for the histochemical and immunohistochemical analysis following I/R, the animals were sacrificed at 0 (sham-operated rats, Sham), 1, 3, 6, 12 and 24 h post-I/R (n  =  5/group) by transcardial perfusion of 0.9% normal saline, followed by 4% paraformaldehyde in 100 mM phosphate-buffered saline. To study the effects of propofol and the autophagy inhibitor 3-methyladenine (3-MA) by histochemical, immunohistochemical and transmission electron microscopic analyses, the rats received an intracerebral ventricular injection of 600 nmol 3-MA (purchased from Sigma, 08592 (Fluka) and dissolved in normal saline by heating the solution to 60–70°C immediately before injection), an intraperitoneal injection of propofol (10, 50, and 100 mg/kg) or an intraperitoneal injection of vehicle (Intralipid, 100 mg/kg) 10 min after I/R and were sacrificed 12 h after I/R. The left femoral artery was cannulated to measure the arterial pH, PaCO_2_, PaO_2_ and blood glucose concentration. These parameters (Table 1) were measured before and during I/R and 60 min after I/R. The body temperature was closely monitored with a rectal probe and maintained at 37.0 ± 0.5°C with a heating pad (Institute of Biomedical Engineering, CAMS, BME-412A Animal Regulator, 308005669) during and after surgery until recovery from anesthesia.

### Transmission Electron Microscopy of Autophagosomes in the Hippocampus after I/R Injury

To observe the time course of the I/R-induced formation of autophagosomes and morphologic changes in the organelles by TEM, the rats were transcardially perfused with phosphate-buffered saline (PBS) (pH 7.4) followed by PBS containing 4% paraformaldehyde (pH 7.4) 1, 3, 6, 12 and 24 h after I/R. To study the effects of the propofol and 3-MA by TEM, the rats were sacrificed 12 h after I/R. The brain tissue samples of 1 cubic millimeter that were removed from the ischemic core of the hippocampus were first immersed in 2.5% glutaraldehyde in 0.1 mol/L phosphate buffer (pH 7.2), post-fixed in 1% osmium tetroxide in 0.1 mol/L phosphate buffer (pH 7.4), dehydrated in graded ethanol series, and flat embedded in Araldite. Ultrathin sections (40–60 nm thick) were placed on grids (200 mesh), and double-stained with uranyl acetate and lead citrate. The sections were observed under a Philips CM-120 electron microscope (Philips).

### Histochemical Analyses

The rats were deeply anesthetized with pentobarbital (25 mg/kg i.p.) and fixed by cardiac perfusion with 4% paraformaldehyde buffered with 0.1 mol/L phosphate buffer (pH 7.2) containing 4% sucrose for light microscopy. For light microscopy, the brain tissues were quickly removed from the rats and further immersed in the same fixative for 2 hours at 4°C. The samples processed for paraffin embedding were cut into 5-µm thick sections using a semi-motorized rotary microtome and placed on silane-coated glass slides. For routine histological studies, the paraffin sections were stained with thionine. For the light microscopy observations, semithin sections were cut 1-µm thick with an ultramicrotome (Ultracut N; Reichert-Nissei, Tokyo, Japan) and stained with thionine.

### Immunohistochemical Analyses

The rats were deeply anesthetized with pentobarbital (150 mg/kg i.p.) and then perfused transcardially with 4% paraformaldehyde in 0.1 mol/L PBS (pH 7.4) 6 or 24 h after I/R. Immunohistochemistry was performed on 18-µm thick cryostat sections. For immunofluorescence labeling, the sections were preincubated for 45 minutes in 15% serum and 0.3% Triton X-100 in PBS and then incubated overnight at 4°C with the primary antibody (Anti-LC3B antibody, polyclonal, Abcam, ab64781) in 1.5% serum and 0.1% Triton in PBS, washed in PBS, and incubated for 2 h in fluorochrome-coupled secondary antibody (FITC, Yeasen, Lot: 94766) at room temperature. The sections were then rinsed in PBS and mounted with FluorSave with the nuclear stain 4′,6′-diamidino-2-phenyl indole dihydrochloride (DAPI) (Sigma, 32670; 5µg/ml). A LSM 510 Meta confocal microscope was used for the confocal laser microscopy. The confocal images were displayed as individual optical sections. For the double labeling experiments, the immunoreactive signals were sequentially visualized in the same section with two distinct filters, with acquisition performed in separated mode. The sections were viewed under high power (200×) with a fluorescence microscope (Eclipse TE 2000, Nikon) with a Nikon digital camera, and the images were visualized in a computer monitor. For the quantification of LC3-II immunostaining, 10 microscopic fields (200× magnification) in each section across ischemic hippocampus regions in the ipsilateral hemisphere were analyzed. Three sections were used for each animal. The number of cells with LC3-II immunoreactivity in each field was counted by an examiner who was blind to the experimental conditions.

### Protein Preparation and Immunoblotting

We deeply anesthetized the rats with an overdose of pentobarbital (100 mg/kg i.p.) and subsequently cut and quickly removed the brain tissues from ischemic hippocampus area and the corresponding area of sham-operated rats. We immediately placed all of the tissue into dry ice-cold collecting tubes and stored them at -80°C until further analysis. The PC12 cells were cultured in 60-mm dishes and harvested and rinsed twice with ice-cold PBS after OGD. We later homogenized these tissue samples and cells in cold Radio Immunoprecipitation Assay lysis buffer (Beyotime Corporation, Nanjing, Jiangsu, China) with a 1% protease-inhibitor cocktail (Sigma-Aldrich, USA), followed by centrifugation at 14,000×*g* for 10 min at 4°C. We determined the protein concentration using a BCA protein assay kit (Beyotime Corporation, China). After heating the aliquots of protein (30 µg) in SDS-PAGE protein loading buffer (Beyotime Corporation, china) at 95°C for 10 min, we separated them on SDS-PAGE gels and transferred the proteins to PVDF membranes (Millipore Corporation, Billerica, MA, USA) for immunoblotting. We incubated the membranes in blocking buffer (5% milk in Tris-buffered saline [TBS] with 0.1% Tween 20) for 1 h at room temperature, followed by an overnight incubation 4°C with primary antibodies against class III PI3K (Monoclonal, Cell Signaling Technology, #3358), Beclin-1 (polyclonal, Cell Signaling Technology, #3738), LC3 (polyclonal, MBL International, PD014), and Bcl-2 (polyclonal, Cell Signaling Technology, #2870). We then washed off the primary antibody three times in TBS, incubated the membranes with horseradish peroxidase-conjugated anti-rabbit IgG antibody (1:5000, Santa Cruz Corporation) for 2 h at room temperature, and washed them three times in TBS. We detected the immunoreactive blots with enhanced chemiluminescence (Amersham Bioscience, Piscataway, NJ, USA) and visualized them on X-ray film (Kodak, Shanghai, China). GAPDH (1:2000; monoclonal, Cell Signaling Technology, #2118) was used as the loading control. The signal intensity of primary antibody binding was quantitatively analyzed with Sigma Scan Pro 5 and was normalized to a GAPDH loading control. The statistical analyses were performed by a one-way analysis of variance (ANOVA) followed by the Tukey test. The differences were considered significant when p< 0.05.

### Statistical Analysis

We analyzed the data using SAS software (Version 8.01, SAS Institute Inc., Cary, NC, USA) and reported the results as the mean±SD. We analyzed the variance in neuronal damage and the number of LC3-II-positive cells in rat hippocampal pyramidal neurons at a given testing time using a one-way ANOVA. For the between-group variance in the ultrastructural changes and the immunoblot analyses of the PC12 cells or rat hippocampal pyramidal neurons at a given testing time, we performed an ANOVA followed by the Tukey test. We considered a result statistically significant when *P*<0.05.
